# MIR600HG suppresses metastasis and enhances oxaliplatin chemosensitivity by targeting ALDH1A3 in colorectal cancer

This article has been retracted.

**DOI:** 10.1042/BSR20200390

**Published:** 2020-04-28

**Authors:** Yi Yao, Nan Li

**Affiliations:** 1 Department of Gastroenterology, Eighth Medical Center of PLA General Hospital, Beijing 100853, China; 2 Medical School of Chinese PLA, Department of Gastroenterology, Chinese PLA General Hospital, Beijing 100853, China

**Keywords:** ALDH1A3, Chemosensitivity, colorectal cancer, Metastasis, MIR600HG

## Abstract

**Background:** Metastasis and chemoresistance indicate a poor prognosis in colorectal cancer (CRC) patients. However, the mechanisms that lead to the development of chemoresistance and metastasis in CRC remain unclear.

**Materials and methods:** We combined clinical and experimental studies to determine the role of MIR600HG in CRC metastasis and chemoresistance. The statistical analysis was performed using GraphPad Prism software, version 8.0.

**Results**: We detected down-regulated expression of long non-coding RNA (lncRNA) MIR600HG in CRC specimens and cell lines compared with normal controls, and the expression level of MIR600HG was inversely correlated with the overall survival of CRC patients. The inhibition of MIR600HG stimulated CRC cell metastasis and chemoresistance. In addition, our data showed that the inhibition of MIR600HG stimulated CRC stemness, while the overexpression of MIR600HG suppressed stemness. Importantly, our animal experiments showed that MIR600HG inhibited tumour formation and that the combination of MIR600HG inhibition and oxaliplatin (Oxa) treatment significantly inhibited tumour growth compared with that with either intervention alone. Furthermore, we demonstrated that MIR600HG exerts its anticancer role by targeting ALDH1A3 in CRC.

**Conclusions:** Our data suggest that MIR600HG functions as a tumour suppressor and that the overexpression of MIR600HG inhibits tumour invasion and enhances chemosensitivity, providing a new strategy for CRC treatment.

## Introduction

Colorectal cancer (CRC) is one of the most common tumours. Approximately 1.2 million patients worldwide are diagnosed with CRC each year, and more than 600000 patients die directly or indirectly from CRC [1]. However, neoadjuvant chemoradiotherapy and surgery greatly improve patient survival time. Early tumour metastasis and chemoresistance are still the main chall enges in the treatment of CRC patients [2–4]. However, the mechanisms that lead to the development of chemoresistance and metastasis in CRC remain unclear.

Cancer stem cells (CSCs) are a small subset of cells within a tumour, and studies show that CSCs are implicated in chemotherapy resistance and metastasis in cancer [5]. CSCs confer high resistance to chemotherapy drugs that are commonly used in the treatment of CRC, including oxaliplatin (Oxa) and 5-fu [6,7]. In addition, studies show that CSCs are able to regenerate all of the cell types in the tumour due to their stem cell-like behavior, resulting in metastatic relapse [7,8]. Therefore, CSCs are important therapeutic targets in cancer. However, the mechanism of CSC regulation in CRC remains unclear.

Long non-coding RNAs (lncRNAs) are non-coding RNA molecules of more than 200 nucleotides in length [9]. They do not encode proteins, but they do regulate gene expression at the transcriptional, post-transcriptional and epigenetic levels and participate in tumour cell proliferation, apoptosis and invasion, metastasis [10]. Additionally, dysregulated expression of lncRNA was demonstrated in CSCs, and such aberrantly regulated lncRNAs are involved in the development of CSCs and the maintenance of stemness [11]. MIR600HG is an RNA gene and is affiliated with the miRNA class. Diseases associated with MIR600HG include pancreatic ductal adenocarcinoma. MIR600HG was then validated to be an independent prognostic predictor for patients with PDAC [12]. Our previous data showed that the decreased expression of MIR600HG was significantly correlated with the overall survival of CRC patients; however, its function and mechanism in CRC remain unclear. Here, we describe a functional role of MIR600HG as a tumour suppressor lncRNA that regulates metastasis, chemoresistance and cancer stemness. Additionally, we identified ALDH1A3 as a target of MIR600HG in CRC.

## Materials and methods

### Cell culture and human specimens

All CRC cells were purchased from the American Type Culture Collection (Manassas, VA) and cultured in DMEM (Sigma–Aldrich, St. Louis, MO) supplemented with 10% foetal bovine serum (HyClone, Logan, UT). Human specimens were obtained from diagnostic biopsies. We selected CRC patients from February 2018 to August 2018. A total of 60 patient specimens and 60 adjacent tissues were used in the present study (Table 1), and informed consent was obtained from each patient who participated in the present study. This research was approved by the Research Ethics Board of the Eighth Medical Centre of PLA General Hospital.

**Table 1:** Characteristics of colorectal carcinoma patients

Characteristics	Variable	Number (%)	*P*-value
Age (years)	Range (means ± SD)	39–76 (60 ± 10)	0.189
Gender	Male	26 (59.1)	0.952
	Female	18 (40.9)	
Family history	No	31 (70.5)	0.432
	Yes	13 (29.5)	
Clinic stage	I	5 (11.4)	0.445
	II	15 (34.1)	
	III	14 (31.8)	
	IV	10 (22.7)	
Pathological type	Adenocarcinoma	30 (68.2)	0.637
	Mucinous carcinoma	14 (31.8)	

### RNA extraction and qRT-PCR

RNA was extracted from cells or tissues using TRIzol reagent (Invitrogen, Carlsbad, CA) and subjected to qRT-PCR. MIR600HG and RNU6 expression was tested by qRT-PCR using a primer set from RiboBio (Guangzhou, China) as a reference [13]. The primer sequence information is defined as follows: MIR600HG forward 5′-TGAGCAGAGTCAAGTGGCAG-3′, reverse 5′-AAAGCCCCATTTCCTAGCCC -3′; U6 forward 5′-GCTTCG GCAGCACATATACTAAAAT-3′; U6 reverse 5′-CGCTTCACGAA TTTGCGTGTCAT-3′. The primer sequences for other genes were defined as follows: ALDH1A3 forward 5′-TGAGTGATTTAGCAGGCTGCA-3′, reverse 5′-TGGCCACATACACCAATAGGTTC-3′; GAPDH forward 5′-GCAGGGGGGAGCCAAAAGGGT-3′, reverse 5′-TGGGTGGCAGTGATGGCATGG-3′. The MIR600HG expression was normalised against RNU6 expression, and ALDH1A3 mRNA expression was normalised against GAPDH. The 2^−ΔΔ*C*_T_^ method was used to analyse the relative fold changes.

### Transwell and osteosphere assays

The Transwell and osteosphere assay protocols were performed as described by Chen et al. [14] and Roscigno et al. [15]. Briefly, 1 × 10^5^ cells in serum-free growth medium were seeded in the upper wells of chambers (12-well plate). The lower wells contained the same medium with 10% serum. After 24 h, the cells that had migrated to the lower side of the chamber were fixed with 2.5% glutaraldehyde, stained with 0.1% Crystal Violet and counted. For the osteosphere assay, 1000 cells were plated in 24-well ultra-low attachment plates in N2B27-defined serum-free medium and cultured for 9 days. Spheres were counted in each plate using a Leica MZ12 inverted microscope.

### Cell viability and apoptosis analysis

After transfection, evaluation of cell proliferation using cell viability was determined using a cell counting kit-8 (CCK-8, Med Chem Express, Monmouth Junction, New Jersey, U.S.A.). Apoptosis assays were performed using the FITC Annexin V Apoptosis Detection Kit I (BD Biosciences) according to the manufacturer’s protocol. Stained cells were analysed by a FACSCalibur flow cytometer (BD Biosciences) [9].

### Luciferase reporter assay

Experiments were performed in triplicate. Luciferase activity was measured using the dual-luciferase assay system (Promega, Madison, WI). The 293T cells were co-transfected with the indicated reporter plasmids and either the pre-MIR600HG or control oligonucleotides (NC) after 48 h of incubation [16]. The 3′-UTR segments of ALDH1A3 that were predicted to interact with MIR600HG were amplified by PCR from human genomic DNA and inserted into the HindIII and SacI sites of the lncRNA Expression Reporter Vector. The primer sequences for amplifying the 3′ UTR of ALDH1A3 are as follows: forward, 5′-AAAGATCCTTTATTAAGCTTTAATAAAATGAGGGCCCGTAACAGAACCAGTG-3′; reverse, 5′-GCGCACTAGTGAGGGAGCTCTTGTGGGATGCGATCTGCAGCTAGGA-3′. For the luciferase reporter experiments, the indicated cells were seeded into 24-well cell culture plates and transfected with the indicated reporter plasmids and either the MIR600HG or negative control oligonucleotides (NC). Following 48 h of incubation, cells were subjected to a luciferase reporter assay.

### Library construction, RNA sequencing and data analysis

First, rRNAs in samples from the control and PM2.5 groups were removed. Then, the libraries for next-generation sequencing were prepared using the TruSeq RNA Sample Prep Kit (Illumina, U.S.A.) according to the manufacturer’s instructions. After enrichment and purification, the libraries were processed for sequencing by Shanghai Origingene Bio-pharm Technology Co., Ltd. (Shanghai, China) according to available protocols. After quality control of the original data, the high-quality sequencing data were compared with the designated reference genome. The expression values were calculated by the StringTie tool, and the tDESeq algorithm was applied to filter the differentially expressed genes.

### Western blot analysis

Cells were lysed, and proteins were isolated. Protein (30 µg) was subjected to Western blotting with anti-ALDH1A3 (Abcam, U.S.A., Cat. No.: ab129815; 1:800), anti-E-cadherin (Abcam, U.S.A.; 1:4000), anti-vimentin (Abcam, U.S.A.; 1:5000), anti-PARP (Abcam, U.S.A.; 1:4000), anti-SOX2 (Abcam, U.S.A.; 1:4000), anti-CD44 (Abcam, U.S.A.; 1:4000) and anti-β-actin (Invitrogen, U.S.A.; 1:10000), and subsequent incubation with secondary antibodies conjugated to horseradish peroxidase (HRP) for 2 h at RT.

### Animal experiments

Animal experiments were conducted using 6-week-old female athymic (nu/nu) mice, and each group included eight mice. A total of 5 × 10^6^ Caco2 cells (stably transfected with a series of lentiviruses were constructed in our laboratory) in 100 µl serum-free medium were injected subcutaneously (s.c.) into each mouse (right back). When the tumours reached ∼50 mm^3^, mice were intraperitoneally (i.p.) injected with oxaliplatin (6 mg/kg body weight). After 3 weeks of drug treatment, mice were killed, and tumour weights were measured. Euthanasia was carried out by CO_2_ in mice when the tumour size reached 1500 mm^3^ (no anaesthetics were used in these experiments). All animal experiments were performed in the Laboratory of PLA General Hospital and were approved by the Research Ethics Board of the Eighth Medical Center of PLA General Hospital (No. 0034/18).

### Statistical analysis

Statistical significance was analysed by unpaired Student’s *t* tests or one-way ANOVA and Duncan’s multiple range tests using the GraphPad Prism software package version 8.0. *P*-values less than 0.05 were considered statistically significant.

## Results

### Down-regulated expression of MIR600HG was associated with poor clinical outcome

Previous studies have shown that some lncRNAs are inversely correlated with CRC progression; MIR600HG expression was significantly decreased in CRC specimens compared with paracancerous specimens in the analysis of data from the TCGA (Figure 1A) and our hospital (Figure 1B). In addition, our clinical data showed that decreased expression of MIR600HG was significantly correlated with the overall survival of CRC patients (Figure 1C). MIR600HG was down-regulated in CRC cell lines compared with the HcoEpiC cell line (Figure 1D). Taken together, these data suggest that MIR600HG may act as a tumour suppressor lncRNA in CRC.

**Figure 1:** Decreased expression of MIR600HG correlates with poor survival of CRC patients (**A**) MIR600HG expression was significantly down-regulated in CRC patients analysis from TCGA database. (**B**) MIR22HG expression was significantly down-regulated in CRC specimens. The expression levels of MIR600HG were measured using qRT-PCR in normal tissue (*n*=50) and tumour tissues (*n*=50). (**C**) Survival rates for CRC patients with low (*n*=20) and high (*n*=20) MIR600HG expression. (**D**) CRC cell lines showed lower expression level of MIR600HG compared with human normal colon epithelial (HcoEpiC) cells. **, *P*<0.01; ***, *P*<0.001.

### MIR600HG inhibits metastasis and chemoresistance in CRC

Then, we investigated the effects of MIR600HG on CRC metastasis and chemoresistance using a CRC cell line transfected with MIR600HG or inhibitor (Figure 2A). We investigated the effects of MIR600HG on the chemotherapy sensitivity of CRC cells. Cell viability and apoptosis analysis results showed that ectopic expression of MIR600HG attenuated CRC cell proliferation and stimulated apoptosis (Figure 2B,D). The combination of MIR600HG and oxaliplatin more significantly accelerated proliferation and stimulated apoptosis compared with single treatment (Figure 2B,D). In contrast, the inhibition of MIR600HG significantly attenuated oxaliplatin-induced CRC cell growth inhibition (Figure 2C). Consistent with cell viability and apoptosis analysis, MIR600HG overexpression significantly enhanced oxaliplatin-induced expression of the pro-apoptotic protein cleaved PARP (Figure 2E). In addition, Transwell experiments showed that the ectopic expression of MIR600HG significantly inhibited CRC cell metastasis, while the inhibition of MIR600HG stimulated CRC cell invasion (Figure 2F). In addition, we examined the effects of MIR600HG on CRC cell EMT because EMT plays an important role in cancer metastasis. Our data show that MIR600HG positively regulates E-cadherin expression in CRC cells but negatively regulates vimentin expression (Figure 2G), suggesting that MIR600HG inhibits EMT in CRC cells. Together, our data suggest that MIR600HG suppresses CRC progression by inhibiting CRC cell invasion and inducing chemoresistance.

**Figure 2:** MIR600HG negatively regulates CRC cells metastasis and chemosensitivity (**A**) Caco2 cells were transfected with negative control oligonucleotide, MIR600HG mimics or MIR600HG inhibitor. After 72 h of transfection, isolated mRNAs were subjected to qRT-PCR. (**B**) MIR600HG enhanced the sensitivity of Caco2 cells to Oxaliplatin treatment. Caco2 cells were transfected with the MIR600HG and treated with or without 0.2 µM Oxaliplatin for 48 h and then subjected to a CCK-8 assay. (**C**) Knockdown MIR600HG expression inhibited the sensitivity of Caco2 cells to Oxaliplatin treatment. Caco2 cells were transfected with the siMIR600HG and treated with or without 0.2 µM Oxaliplatin for 48 h and then subjected to CCK-8 assay. (**D**) The MIR600HG overexpression enhanced Oxaliplatin-induced apoptosis in Caco2 cells. MIR600HG overexpression Caco2 cells were treated with DMSO or 0.2 μM Oxaliplatin for 24 h and analysed with flow cytometry. (**E**) MIR600HG stimulates Oxaliplatin-induced expression of cleaved- and total-PARP in CRC cells. Caco2 cells were transfected with the MIR600HG or treated with 0.2 µM Oxaliplatin for 48 h, and then subjected to Western blotting. (**F**) MIR600HG negatively regulates Caco2 cell metastasis. After 24 h of transfection, cells were subjected to an invasion assay. (**G**) MIR600HG inhibited EMT in CRC cells. Caco2 cells were transfected with negative control oligonucleotides, MIR600HG mimics or MIR600HG inhibitor. After 72 h of transfection, cells were subjected to Western blot analysis for the detection of the expression of the indicated proteins. NC, negative control oligonucleotides; mimics, MIR600HG mimics; inhibitor, MIR600HG inhibitor; Oxa, Oxaliplatin; *, *P*<0.05; **, *P*<0.01.

### RNA transcriptome sequencing analysis of the MIR600HG downstream regulatory pathway

We constructed MIR600HG-overexpressing Caco2 cell lines for sequencing, with normal controls included. PCA shows that the two groups of samples are almost completely different (Figure 3A), and the heat map also shows that there is a large difference between the groups (Figure 3B). A volcano map (Figure 3C) was generated for the two groups of samples (tools, R language limma package). The volcano map showed that compared with the low miR600HG expression group, the high miR600HG expression group had a large number of down-regulated proteins. Enrichment analysis revealed the top 30 signalling pathways related to MIR600HG expression (Figure 3D), which suggested that MIR600HG may affect the process of colon cancer by affecting the pluripotency of colon cancer cells.

**Figure 3:** Analysis of MIR600HG downstream regulatory pathway We constructed MIR600HG overexpressing Caco2 cell lines for RNA sequencing with normal controls. (**A**) PCA analysis can find that the two groups of samples are almost completely different. (**B**) The heat map also shows the sample. There is a large difference between them. (**C**) The volcanic map was performed on the two groups of samples (tools, R language limma package). The volcano map showed that compared with the miR600HG low expression group, the miR600HG high expression group had a large number of proteins with low expression. (**D**) KEGG Enrichment analysis, taking the first 30 signal pathways as a map, suggesting that MIR600HG may affect the process of colon cancer by affecting the pluripotency of colon cancer cells.

### ALDH1A3 is a target of MIR600HG

To investigate how MIR600HG regulates metastasis and chemoresistance in CRC, we searched for candidate target genes of MIR600HG (mirdb.org) and identified ALDH1A3 as a candidate of MIR600HG (Figure 4A). Thus, we chose to further study ALDH1A3. To investigate whether MIR600HG is involved in ALDH1A3 regulation, Caco2 cells were transfected with MIR600HG or inhibitor. After 72 h of transfection, ALDH1A3 expression was measured using qRT-PCR and Western blot. Our experimental results showed that ALDH1A3 expression was significantly up- or down-regulated by the inhibition or ectopic expression of MIR600HG, respectively, in CRC cells at both the mRNA and protein levels (Figure 4B,C). Furthermore, we verified that MIR600HG directly targeted the 3′ UTR of ALDH1A3 by using a luciferase reporter assay (Figure 4D). Consistent with the *in vitro* results, the clinical sample analysis results also showed an inverse association between ALDH1A3 and MIR600HG in CRC specimens (Figure 4E). These findings indicated that MIR600HG inhibits ALDH1A3 mRNA and protein expression by directly targeting its 3′ UTR.

**Figure 4:** MIR600HG targets ALDH1A3 (**A**) The MIR600HG seed sequence is complementary to the 3′ UTR of ALDH1A3. (**B,C**) MIR600HG inhibited ALDH1A3 mRNA and protein expression. After 72 h transfection of MIR600HG and siMIR600HG, using qRT-PCR and Western blot measurement. (**D**) Activity of the luciferase gene linked to the 3′ UTR of ALDH1A3. The luciferase reporter plasmids of wild-type (WT) or mutated 3′ UTR sequences of ALDH1A3 (MT) were transfected into HEK-293 cells with or without the MIR600HG. (**E**) The expression levels of ALDH1A3 and MIR600HG showed a negative correlation in CRC patients. Tumour samples were obtained from ten patients with CRC, and the expression of ALDH1A3 and MIR600HG were measured by RT-qPCR. NC, negative control inhibitor, MIR600HG inhibitor; ns, no significance; **, *P*<0.01.

### MIR600HG inhibits cancer stemness via ALDH1A3 in CRC

Previous studies have shown that stem cells cause metastasis and chemoresistance in cancers; ALDH1A3 plays a key role in CSC maintenance and is closely associated with cancer metastasis and chemoresistance [17–19]. We investigated whether MIR600HG is involved in CSC regulation in CRC. As expected, the osteosphere assay showed that the inhibition of MIR600HG significantly increased osteosphere numbers, while the overexpression of MIR600HG reduced osteosphere numbers compared with those in the control (Figure 5A). Consistent with sphere formation results, Western blot results also showed that the overexpression of MIR600HG significantly inhibited the expression of CSC marker proteins, including SOX2 and CD44 (Figure 5B). However, increasing ALDH1A3 expression reversed the inhibition of CSC marker protein expression by MIR600HG (Figure 5B). These data suggest that MIR600HG exerts its anticancer effects partially due to the inhibition of cancer stemness in CRC.

**Figure 5:** MIR600HG negatively regulates CRC stemness (**A**) The inhibition of MIR600HG stimulated osteosphere formation in Caco2 cells, whereas the overexpression of MIR600HG inhibited osteosphere formation. (**B**) MIR600HG negatively regulated CSC marker protein expression. Caco2 cells were transfected with the MIR600HG and siMIR600HG. After 72 h of transfection, cells were subjected to Western blot analysis. NC, negative control oligonucleotides; inhibitor, MIR600HG inhibitor; *, *P*<0.05; **, *P*<0.01.

### ALDH1A3 is a functional target of MIR600HG that modulates CRC metastasis and chemoresistance

Finally, we investigated whether ALDH1A3 is involved in the MIR600HG-mediated regulation of metastasis and chemoresistance. The cell viability analysis results showed that the overexpression of ALDH1A3 restored the cell proliferation inhibited by MIR600HG (Figure 6A); in contrast, silencing of ALDH1A3 suppressed MIR600HG inhibition-induced cell growth (Figure 6B). Consistent with these results, the apoptosis analysis showed that the overexpression of ALDH1A3 attenuated MIR600HG-induced cell apoptosis (Figure 6C). In addition, Transwell experiments showed that the overexpression of ALDH1A3 attenuated the MIR600HG-induced metastasis effect (Figure 6D). Together, our data suggest that MIR600HG regulates metastasis and chemoresistance via ALDH1A3 in CRC.

**Figure 6:** ALDH1A3 is a functional target of MIR600HG that modulates CRC metastasis and chemosensitivity of Oxaliplatin (**A**) The cell viability analysis results show that the overexpression of ALDH1A3 restored the cells viability inhibited by MIR600HG and decreased chemosensitivity of Oxaliplatin. (**B**) Silencing of ALDH1A3 suppressed MIR600HG inhibition-induced cells viability and increased chemosensitivity of Oxaliplatin. (**C**) The apoptosis analysis ALDH1A3 overexpression attenuated the MIR600HG induced cell apoptosis, decreased chemosensitivity of Oxaliplatin. (**D**) Transwell experiments showed that the overexpression of ALDH1A3 attenuated the MIR600HG-induced metastasis effect. NC, negative control oligonucleotides; inhibitor, MIR600HG inhibitor; ALDH1A3: ALDH1A3 plasmid; siALDH1A3, siRNA of ALDH1A3; *, *P*<0.05; **, *P*<0.01.

### MIR600HG significantly inhibits tumorigenesis and chemoresistance *in vivo*

As shown in the animal experiment, tumour volume and weight (Figure 7A,B) was significantly decreased in the MIR600HG overexpression group compared with the control group. Additionally, we detected the CSC marker CD133 in tumour tissues, and the data showed that the groups treated with MIR600HG had a significantly reduced CD133 mRNA level compared with that in the groups that were not treated with MIR600HG (Figure 7C). Consistent with these results, Ki-67 IHC assay (Figure 7D) results clearly showed that combined oxaliplatin treatment and MIR600HG inhibition suppressed cell proliferation more potently and significantly than the single treatments. Taken together, these data suggest that MIR600HG is essential to blocking tumour formation and improving chemosensitivity (Figure 7E).

**Figure 7:** MIR600HG overexpression in combination with Oxaliplatin inhibits tumour relapse (**A,B**) Tumour volume and weight in xenografts treated with Oxaliplatin, MIR600HG or both at days 29, 32 and 36. Caco2 cells and injected s.c. into nude mice (*n*=9/group, 1 × 10^4^ cells/mouse). (**C**) The level of CD133 mRNA derived from xenograft model tumour analysis by RT-PCR. (**D**) Ki-67 immunohistochemistry assay show that combination of MIR600HG inhibition and Oxaliplatin treatment more significantly inhibits cell proliferation in xenograft tumour. (**E**) A schematic model of MIR600HG target ALDH1A3 inhibited CRC metastasis and chemosensitivity. NC, negative control oligonucleotides; inhibitor, MIR600HG inhibitor; Oxa, Oxaliplatin. *, *P*<0.05; **, *P*<0.01.

## Discussion

The occurrence of chemoresistance and metastasis indicates poor survival in CRC patients [10]. In the present study, we provide insight into the biological effects of MIR600HG in CRC metastasis and chemoresistance by using a series of experiments. Here, we found that increased expression of MIR600HG significantly correlated with good clinical outcomes in CRC patients. This result is consistent with Song et al.’s reports that lncRNA MIR600HG is associated with poor prognosis in patients with PDAC [12]. In addition, our *in vitro* study showed that the overexpression of MIR600HG enhanced the chemosensitivity of CRC cells to anticancer drugs and inhibited CRC cell invasion. In contrast, the inhibition of MIR600HG promoted CRC cell invasion and decreased chemosensitivity. These findings showed that MIR600HG functions as a tumour suppressor and that targeting MIR600HG may be a novel strategy for suppressing CRC metastasis and enhancing chemosensitivity.

We further clarified the anti-CRC mechanism of MIR600HG. We used a series of experiments to identify ALDH1A3 as a target gene of MIR600HG in CRC. Our data showed that ALDH1A3 expression was up- or down-regulated in CRC cells by the inhibition or ectopic expression of MIR600HG, respectively. Previous studies have shown that ALDH1A3 is a CSC marker and plays an important role in CSC regulation [20,21]. Accumulated evidence has shown that increased cancer stemness can stimulate cancer metastasis and induce chemoresistance [22–24]. MIR600HG may regulate CSCs by targeting ALDH1A3, so we investigated the CSC regulation mechanism of MIR600HG in CRC. Our data showed that the inhibition of MIR600HG stimulated CRC stemness. More importantly, our experiments showed that the overexpression of MIR600HG significantly suppressed cancer stemness and reduced CSC populations in tumour tissues, suggesting that MIR600HG plays an anticancer role partially by inhibiting CRC stemness. In addition, our data showed that the restoration of ALDH1A3 blocked the MIR600HG overexpression-induced inhibition of cancer stemness. In general, these data suggest that MIR600HG inhibits CRC metastasis and chemoresistance through the inhibition of cancer stemness by targeting ALDH1A3.

In summary, we combined clinical and experimental studies to establish a role for MIR600HG in CRC metastasis and chemoresistance. The overexpression of MIR600HG dramatically enhances the sensitivity of CRC cells to chemotherapy and inhibits CRC metastasis through suppressing CRC stemness by targeting ALDH1A3. Our findings may also help develop potential therapeutics for the treatment of CRC metastasis and chemoresistance.

## Data Availability

All data generated or analysed during the present study are included in this published article.

## Abbreviations

5-fu: 5-fluorouracil
ALDH1A3: aldehyde dehydrogenase family 1 member A3
CRC: colorectal cancer
CSC: cancer stem cell
EMT: epithelial-mesenchymal transition
IHC: immunohistochemistry
LncRNA: long non-coding RNA
MIR600HG: lncRNAs MIR600HG
Oxa: oxaliplatin
PARP: poly-ADP-ribosyl transferase polymerase
PCA: principle component analysis
PDAC: pancreatic ductal adenocarcinoma
RT: reverse transcription
SOX2: transcription factor SOX-2
